# Protective Effect of Galangin Methylation Modification Based on Cell Imaging on Inflammatory Lung Injury and Its Molecular Mechanism

**DOI:** 10.1155/2022/7511345

**Published:** 2022-08-16

**Authors:** Ke Hu, Yuxian Li, Ling Jin, Yuefu Chen, Lijun Chen, Yingjun Zhang, Minjiang Huang, Yan Ding, Huiming Yin, Minghua Liang, Bifeng Tan

**Affiliations:** ^1^Medical College, Hunan University of Medicine, Jinxi South Road No.492, Huaihua 418000, Hunan, China; ^2^Department of Respiratory and Critical Care Medicine, First Affiliated Hospital, Hunan University of Medicine, Yushi Road No.225, Huaihua 418000, Hunan, China; ^3^Department of Pediatrics, First People's Hospital of Huaihua, Jinxi South Road No.144, Huaihua 418000, Hunan, China; ^4^Department of Cardiology, First Affiliated Hospital, Hunan University of Medicine, Yushi Road No.225, Huaihua 418000, Hunan, China

## Abstract

**Background:**

Recently, inflammation has become a major threat to human health. Studies have confirmed that some Chinese traditional medicine ingredients may effectively interfere with the expression of inflammatory mediators through epigenetic modification, showing a great potential of the application.

**Objective:**

To investigate the role of the PPAR/DNMT3A pathway in the reversal of galangin-mediated inflammatory lung injury, promote the development of new anti-inflammatory drugs, reduce the side effects of chemical synthetic drugs on the body, and prove the effectiveness and safety of galangin in inhibiting inflammatory response and injury.

**Methods:**

120 rats were randomly divided into 6 groups: (Group 1) LPS group; (Group 2) LPS + galangin group; (Group 3) LPS + galangin +  GW9662 group; (Group 4) LPS + galangin + DNMT3A siRNA group; (Group 5) LPS + galangin + siRNA negative group; (Group 6) control group. The model of inflammatory lung injury was established by intrathecal instillation of LPS in the first five groups and NS in the control group. SD survival rate was recorded every 24 hours after modeling, lasting for 168 hours. The lung tissues were taken 168 hours after the establishment of the model. The pathological morphology of lung tissue was observed after the staining under the light microscope, and the lung dry/wet weight ratio was calculated after drying. After NS was perfused into lung tissue, the lavage fluid was collected and the levels of IL-6 and TNF-a were measured by ELISA. The contents of PPAR, DNMT3A, phosphorylated p65, and ERK in monocytes were detected by the WB method, and the binding contents of p65 and AP-1 in the promoter regions of IL-6 and TNF-a genes were detected by the Chip-qPCR method.

**Results:**

Intraperitoneal injection of galangin could inhibit the synthesis of alveolar inflammatory factors (TFs) in the SD model of lung injury induced by LPS, reduce the degree of pathological injury of lung tissue, and improve the survival rate of the SD model. GW9662 can completely reverse the protective effect, while DNMT3A interference can only partially block its protective effect. In addition, galangin could significantly inhibit the LPS-induced expression of p65 and AP-1 in alveolar monocytes and their binding content in the promoter region of inflammatory genes by activating PPAR/DNMT3A pathway. GW9662 could completely reverse the inhibitory effect of galangin. DNMT3A interference could restore the binding content of transcription factors at the promoter of the inflammatory gene but had no significant effect on its synthesis.

**Conclusion:**

Galangin can interfere with the binding of transcription factors to inflammatory gene promoters through the methylation modification induced by PPAR/DNMT3A pathway, so as to inhibit the synthesis of inflammatory molecules and reverse inflammatory lung injury.

## 1. Introduction

Acute lung injury (ALI) refers to the injury of alveolar epithelial cells and capillary endothelial cells caused by various harmful factors, resulting in diffuse pulmonary interstitial and alveolar edema, leading to acute hypoxic respiratory insufficiency, which will develop into acute respiratory distress syndrome (ARDS) [1]. At present, glucocorticoid is the main clinical intervention for ALI, although it is effective and can easily cause side effects after long-term use [2]. It was found that ACA (acetoxychavicol acetate) compounds in rhizomes of *Alpinia officinale* are effective inhibitors of NLRP3 inflammatory bodies, which could prevent NLRP3-related inflammatory diseases [3]. In addition, ACA is a natural compound in the roots of tropical ginger galangal, which is beneficial to inflammatory lung injury. Thus, seeking anti-inflammatory drugs with less toxic side effects has become essential, with flavonoids receiving gradual attention. Flavonoid drugs generally possess a peroxisome proliferator-activated receptor (PPAR) agonistic activity [4, 5], closely associated with inflammatory factor synthesis inhibition. Among them, galangin has proven to affect the progression of inflammatory diseases like ulcerative colitis and atherosclerosis in animal models, owing to its potent PPAR agonistic activity [6, 7]. Early in vitro experiments confirmed that galangin could promote the PPAR binding to the methyltransferase DNMT3A in RAW246.7 nuclei and induce DNMT3A activation, facilitating the methylation modification of inflammatory gene promoter fragments to inhibit the expression of inflammatory molecules. Therefore, we speculate that PPAR/DNMT3A pathway may mediate the intervention of galangin on inflammatory diseases. In order to test this hypothesis, we established the inflammatory lung injury model of SD rats by intratracheal instillation of LPS, confirmed that galangin could reverse the process of inflammatory lung injury through the PPAR/DNMT3A pathway, and discussed its specific protective mechanism. The results of this study could provide a reliable theoretical basis for the clinical application of the drug.

Our preliminary research proved that inducing the intranuclear synthesis of PPAR and stimulating its activity is essential to inducing the anti-inflammatory role of galangin. PPAR activation can lead to the inhibited synthesis of classic inflammatory TFs like nuclear factor *κ*B (NF-*κ*B) and extracellular receptor-activated kinases (ERKs), associated with the suppressed expression of inflammatory factors (such as IL-6 and TNF-*α*) [8, 9]. Furthermore, the research found that PPAR activation could stimulate histone deacetylase 1 (HDAC1) activity, leading to deacetylation of histones bound to the inflammatory gene promoters. The latter blocks TF binding to the promoters, thereby suppressing the inflammatory gene expression. This is consistent with several reports suggesting that acetylation modification is involved in inflammatory disorder development [10, 11]. To summarize, we speculate that the pharmacological effects following PPAR activation involve epigenetic modification.

Furthermore, studies also confirmed that the stimulation of deacetylation modification may only be part of the effect after PPAR activation. In the epigenetic modification mechanism of regulating gene expression, methylated modification is more common. Some studies have reported that abnormal methylation is involved in the occurrence and progression of specific diseases. For example, in monocytes of atherosclerotic (as) animals, the methylation level of multiple CpG sites in the core regulatory region of the TLR4 promoter decreased, which was negatively correlated with the expression of TLR4 mRNA [12]. In addition, the expression levels of histone 3-lysine-4-methyltransferase (MLL2) and DNA methyltransferase 1 (DNMT1) in vascular tissues near as lesions were higher than those in normal vascular wall tissues [13]. In addition, the level of methylated H3K27 in advanced atherosclerotic plaque increased significantly, and the expression of histone methyltransferase G9a and DNMT1 increased [14]. Besides, the methylation degree of H3K27 and membrane integrin ABCA1 promoter could be reduced by transfecting macrophages with the interference fragment of enhancer of zeste homolog 2 (EZH2). Thus, elevating ABCA1 expression to transport lipids out of cells could be a novel direction for as treatment [15]. In addition, foam cell formation and inflammatory molecule synthesis induced by oxidized low-density lipoproteins are associated with methylation integration [16]. Abnormal methylation has been confirmed to be associated with tumor occurrence in the head, neck, and digestive tract [17, 18]. Research claims that the level of abnormal methylation in peripheral blood cells can be a novel marker for predicting tumorigenesis risk [19]. Based on the abovementioned research, abnormal methylation could be involved in various clinical diseases' occurrence and progression.

By employing the co-immunoprecipitation technique, we further demonstrated that galangin could promote the binding of PPAR and DNMT3A in RAW246.7 nuclei in a dose-dependent manner [20]. DNMT3A, as a major CpG methyltransferase, consists of an N-terminal binding domain and a C-terminal with transmethylation activity [21], regulating the target genes expression by quickly converting cytosine into 5-methylcytosine [22]. Galangin was found to promote the methylation of promoter CpG sites of IL-6, a key inflammatory gene, via the PPAR/DNMT3A pathway, thereby inhibiting IL-6 expression [23]. In summary, methylation induction should be part of the mechanism, wherein galangin intervenes to synthesize inflammatory mediators. Moreover, the PPAR/DNMT3A pathway is also highly likely to mediate the reversal of inflammatory injury by galangin. Verification of the abovementioned hypothesis will further prove the anti-inflammatory value of galangin.

## 2. Materials and Methods

### 2.1. Materials

One hundred twenty clean male SD rats (8–10 weeks old, weight 250 ± 25 g) were purchased from the Laboratory Animal Center of Central South University (License No.: SYKK [X]2016–0002), approved by the Ethics Committee of Hunan University of Medicine. Lenti-DNMT3A and negative interfering lentiviral vector were constructed by Wuhan Bioengineering Technology Co., Ltd. Pure galangin extract (molecular formula: C16H14O4) was purchased from Zelang Biotechnology Co., Ltd., Nanjing. RAW246.7 was purchased from Hwatao Biopharm Co., Ltd., Nanjing, while GW9662 (PPAR antagonist, molecular formula: C13H9CN2O3), PCR Buffer, dNTP, and DNA marker were from Sangon Biotech Co., Ltd., Shanghai. DNA Ladder (100 bp) and Chip assay kit were purchased from Promega, the USA, and PPAR, DNMT3A, p65, and AP-1 monoclonal primary antibodies were purchased from BioDev-Tech. Co., Ltd. IL-6 and TNF-a ELISA kits used were from HY-Tech Biomedical Technology Co., Ltd., Beijing.

### 2.2. Methods

#### 2.2.1. Establishment of the Inflammatory Lung Injury Model and Animal Grouping

A total of 120 SD rats were divided into six groups according to a random number, namely, control group, LPS group, LPS + galangin group, LPS + galangin + GW9662 group, LPS + galangin + DNMT3A interference group, and LPS + galangin + negative interference group (*n* = 20 per group). The specific steps of lung injury model preparation were based on literature [24], where the LPS dosage of the model group was 0.5 mg/kg and the tracheas of the control group were instilled with the same volume of NS as the model group. Both galangin (50 mg/kg) and GW9662 (100 mg/kg) were injected intraperitoneally 2 h following LPS administration. Intravenous bolus injection was given to the DNMT3A and negative interference groups at the tail edge at 108 TU/200 *μ*L per rat, 4 h following LPS administration. After model establishment, the survival ratios of rats in various groups were recorded at 24 h intervals and completed at 168 h. The chest was opened after anesthetization with buprenorphine (0.05 mg/Kg).

#### 2.2.2. Determination of IL-6 and TNF-a in Bronchoalveolar Lavage Fluid (BALF)

The unilateral proximal bronchus (except for the lung tissues) was ligated, and a 5# scalp needle was pierced into the bronchus and fixed, keeping it away from the lung tissues. Sterilized PBS (at 4°C) was infused slowly along the needle until the entire lung was slightly recruited. The PBS was withdrawn after 30 sec. This process was repeated several times to recover BALF. The erythrocytes were precipitated by 5% hetastarch, and the supernatant was collected, centrifuged at 4°C, 3000 rpm for 5 min, to collect the cell pellets and supernatant. The mass concentrations of IL-6 and TNF-a in the supernatant were assayed using ELISA as per the manufacturer's instructions. The standard solution's absorbance was measured at 490 nm with an ELISA reader, and standard curves were plotted, based on which the mass concentrations were read.

#### 2.2.3. Calculation of Lung Tissue Dry/Wet Weight Ratio

On the other side, the upper lung lobe was isolated, placed in a dry glass tube after removing surface water with filter paper, accurately weighed on an electronic balance, and then placed at a constant temperature oven at 100°C for 12 h, followed by withdrawal and weighing. The ratio of masses after to before incubation was regarded as the dry/wet weight ratio.

#### 2.2.4. Pathomorphological Evaluation of Lung Tissues

On the other side, the lower lung lobe was fixed in 4% paraformaldehyde for 24 h, dehydrated with 300 mL/L sucrose solution, embedded in paraffin, and prepared into 5 *μ*m tissue sections. The tissue sections were stained with conventional HE and observed under an optical microscope.

#### 2.2.5. Western Blotting of PPAR, DNMT3A, p65, and AP-1 Contents in BALF Monocyte Nuclei

The collected cell pellets were suspended in PBS, added to a lymphocyte separation medium, and incubated for 30 min. The ivory middle layer (primarily monocytes) was carefully pipetted, incubated with RPMI-1640, and adjusted for cell density in a 96-well plate. About 106 viable normal cells from each group were selected and sequentially subjected to nucleoprotein extraction, membrane transfer, sealing, and addition of labeled PPAR, DNMT3A (1 : 1000), p65, AP-1 (1 : 2000) primary antibody, and HRP-labeled secondary antibody (1 : 1000), as well as developed according to the Molecular Cloning: A Laboratory Manual. The optical density of target bands was analyzed using AlphaEase FC version 4, and the result was expressed as the gray ratio of target protein/internal reference.

#### 2.2.6. Chip-qPCR Assay of p65 and AP-1 Binding Capacities in IL-6 and TNF-a Gene Promoter Regions

The first 3000 bp fragments of transcription start (TSS) point of rat IL-6 and TNF-a genes were obtained on the Genomic Sequence browser of the UCSC website, which were input into the Cpgplot program to confirm that both 300–1300 bp upstream of IL-6 TSS and 250–800 bp upstream of TNF-a TSS met the CpG island criteria. The abovementioned two confirmed CpG island regions were input into Alibaba 2.0 database for separate analysis of transcription factor (TF) binding sites, confirming the presence of p65 and AP-1 binding sites, respectively (see Figures 1(g) and 1(i)). Furthermore, 10^6^ viable normal monocytes were collected and subjected to Chip-qPCR as per the following steps: (1) Protein-DNA crosslinking and cell lysis: cells were fixed in 1% formaldehyde solution, washed with PBS, centrifuged to remove the supernatant, and added with 1 mL of protease inhibitor-containing SDS lysate. (2) Ultrasonic shearing of chromatin was performed at 100 W for 10 s per time, 5 times in total. The chromatin in cell lysate was sheared at 30 s intervals and centrifuged at 4°C to retain the supernatant. (3) Co-immunoprecipitation: the protein G-Sepharose beads were added to the sonicated lysate for preclearing, and TF monoclonal antibody (10 *μ*g/tube) was added to the remaining supernatant and incubated on a shaker at 4°C for 12 h. The immunocomplex was captured by adding protein G-Sepharose beads and sequentially washing with different concentrations of salt and lithium chloride after supernatant removal and centrifugation. (4) Protein-DNA de-crosslinking: after incubation with 5 mol/L NaCl solution in a 65°C water bath overnight, DNA was recovered from the spin column. (5) Real-time PCR of the relative contents of p65 and AP-1 bound to IL-6 and TNF-a CpG islands. Initially, PCR primers were designed according to the following criteria: (1) all the amplified regions should be located within the CpG islands; (2) all the upstream and downstream primers should cover at least one TF binding site. In addition, a pair of upstream and downstream sequences, used for amplifying the second intron of IL-6, was designed as a reference.

#### 2.2.7. Statistical Analysis

All the quantitative data were expressed as mean ± standard deviation. Multigroup comparison was performed by one-way ANOVA, pairwise comparison was done by the least significant difference (LSD) method, and survival rates were compared using Kaplan–Meier analysis. SPSS 19.0 was used for statistical analysis, where *P* < 0.05 was considered statistically significant.

## 3. Results

### 3.1. Galangin Attenuates LPS-Induced Lung Injury, While GW9662 and DNMT3A Interference Reverse This Effect

Table 1 lists the relevant sequences designed according to the abovementioned principles. The reaction program consisted of a total of 40 cycles at 94°C for 5 s and 60°C for 30 s. Semiquantitative results were obtained by electrophoresis, which represent the relative binding capacities of p65 and AP-1 in the IL-6 and TNF-a promoter regions.

#### 3.1.1. BALF IL-6 and TNF-a Levels in Various Groups

The ELISA results of IL-6 and TNF-a levels in BALF are presented in Figures 2(a) and 2(b), respectively. The LPS group exhibited significantly higher counts of inflammatory cells in BALF than in the NS group and markedly higher IL-6 and TNF-a levels. Galangin could inhibit the LPS-induced inflammatory cell counts and inflammatory mediator concentrations. In addition, the inhibitory effect of galangin could be entirely reversed by the PPAR antagonist GW9662, while DNMT3A interference could only partially reverse such inhibitory effect on the inflammatory mediator synthesis.

#### 3.1.2. Lung Tissue Dry/Wet Weight Ratio of Various Groups

Figure 2(c) depicts the dry/wet weight ratios of rat lung tissues of each group. The variation trends were consistent with the inflammatory cell counts and inflammatory mediator concentrations in BALF. In other words, the dry/wet weight ratio was significantly lowered in the LPS group, while galangin could restore this ratio of lung tissues. However, this restoration could also be reversed fundamentally by GW9662 and partially by DNMT3A interference.

#### 3.1.3. Pathomorphological Observation of Lung Tissues in Various Groups

The HE staining results of lung tissue sections are displayed in Figure 2(d) for each group. The NS group's alveolar walls were thin and smooth, with no apparent cell exudation in the alveolar cavity or lung interstitium. In contrast, the LPS group exhibited prominent infiltration of inflammatory cells into the alveolar cavity and lung interstitium, with a severely damaged alveolar wall structure. Galangin could repair the LPS-induced pathological changes in the lung tissue structure, although such effect was also reversible by GW9662 and DNMT3A interference. However, negative interference did not affect the protective effect of galangin.

#### 3.1.4. Survival Rates of SD Rats in Various Groups

Intergroup survival was compared using Kaplan–Meier survival analysis and is depicted in Figure 2(e). All rats in the NS group survived 168 h after model establishment. The lowest survival rate was found in the LPS group (10%), which could be restored to 65% by intraperitoneal injection of galangin. GW9662 could block the survival restoration effect of galangin in SD rats. DNMT3A interference could also partially reverse the survival restoration effect of galangin in SD rats. However, negative interference did not affect such restoration effect of galangin.

### 3.2. PPAR/DNMT3A Pathway Mediates the Inflammatory Molecule Synthesis Inhibition by Galangin in Rat Monocytes

#### 3.2.1. DNMT3A, a Downstream Molecule following PPAR Activation

Western blotting (WB) was employed to detect the PPAR and DNMT3A contents in BALF monocyte nuclei in each group to verify the upstream and downstream relationship between PPAR and DNMT3A, as depicted in Figures 1(a)–1(c). The intranuclear PPAR and DNMT3A contents of the LPS group were lower than those of the NS group, while galangin could restore the expression of both PPAR and DNMT3A. GW9662 was shown to block the promotion of DNMT3A expression by galangin, while DNMT3A interference was unable to influence the high PPAR expression. Thus, DNMT3A could be a downstream molecule following PPAR activation induced by galangin.

#### 3.2.2. Methylated Modification Does Not Involve TF Synthesis

WB technique was employed to assay the levels of classic inflammatory TFs (p65 and AP-1) in BALF monocyte nuclei and is presented in Figures 1(d)–1(f). LPS could promote the intranuclear TF synthesis compared to the NS group, while galangin could inhibit the synthesis induced by LPS. Furthermore, the analysis revealed that GW9662 could restore the TF synthesis, while DNMT3A interference had no restoration effect on the galangin-induced inhibition of TF synthesis. To sum up, although PPAR activation directly inhibited the classic TF synthesis, DNMT3A, a downstream molecule of PPAR, was not directly involved.

#### 3.2.3. Methylated Modification Interferes with Inflammatory Activation by Hindering TF Binding to Inflammatory Gene Promoters

In order to further clarify the specific molecular mechanism of methylation modification interfering with inflammatory expression, the content of phosphorylated TFs bound to inflammatory gene IL-6 and TNF-a promoter CpG island in different groups of monocytes was analyzed by Chip-qPCR. The semiquantitative PCR results of amplified regions were used to represent the relative binding capacities. p65 binding to IL-6 CpG island is presented in Figures 1(g) and 1(h), and AP-1 binding to TNF-a is given in Figures 3(i) and 3(j). LPS could significantly promote the binding of phosphorylated TFs to IL-6 and TNF-a CpG islands compared to the NS group. However, galangin inhibited the promotion of bindings by the LPS mentioned above. Furthermore, the analysis showed that GW9662 completely restored the binding of TF to the inflammatory gene CpG island. In addition, DNMT3A interference also partially restored the binding of TF to the inflammatory gene CpG island. Thus, the PPAR activation-induced methylated modification was likely to interfere with inflammatory mediators' expression by preventing classic TFs from binding to the CpG islands of inflammatory gene promoters, thereby reversing the inflammatory injury.

## 4. Discussion

Acute lung injury (ALI) is the injury of alveolar epithelial cells and capillary endothelial cells caused by various direct and indirect injury factors, resulting in diffuse pulmonary interstitial and diffuse pulmonary interstitial and alveolar edema and acute hypoxic respiratory insufficiency. Despite constant research, the prognosis of ALI remains unsatisfactory due to the lack of drugs that can effectively inhibit the inflammatory mediator production without causing side effects [25]. At present, the research is gradually focusing on the anti-inflammatory TCM constituents, of which galangin, a flavonoid drug, is a typical representative. Hence, it is imperative to explain the anti-inflammatory mechanism of galangin comprehensively. *Alpinia officinale* has been recorded in many pharmacopoeias in ancient China, such as the compendium of Materia Medica and Chinese Pharmacopoeia. *Alpinia officinale* has a good inhibitory effect on inflammatory lung injury. ACA compounds extracted from *Alpinia officinale* rhizome can prevent NLRP3-related inflammatory diseases and have the characteristics of antimicrobial, antiallergic, and anticancer properties.

In the present experiment, we initially established an SD rat model of inflammatory lung injury by tracheal instillation of LPS. The model preparation was ideal by measuring indices such as BALF IL-6 and TNF-a levels, lung tissue dry/wet weight ratio, pathological alteration, and survival curve and comparison with the NS group. Intraperitoneal injection of galangin can remarkably inhibit the LPS-induced synthesis of IL-6 and TNF-*α*, the change in lung tissue dry/wet weight ratio, and the disruption of lung tissue structure, improving the survival rate of rats with inflammatory lung injury. When the PPAR antagonist, GW9662, is used in combination or DNMT3A interference is adopted, the protective effect of galangin is completely or partially reversed. To further verify the specific roles of PPAR and DNMT3A activation in the intervention of inflammation, we proved through an in vitro experiment that DNMT3A is a downstream molecule of PPAR. GW9662 can completely block the galangin inhibitory effect on the expression of classic inflammatory TFs (p65 and AP-1), while the DNMT3A interference shows an insignificant impact on the synthesis of TFs. According to the CpG islands and TF binding sites present at the murine IL-6 and TNF-*α* promoters, Chip-qPCR was used to assay the TF levels in the IL-6 and TNF-*α* promoter CpG islands. It revealed that the DNMT3A interference could partially restore the galangin-induced decrease in TF binding capacities, albeit less significant than the GW9662 group. Based on the abovementioned experiment, we speculate that at least two types of mechanisms are involved in the anti-inflammatory effect of galangin. Firstly, PPAR activation directly inhibited the synthesis of classic inflammatory TF. Besides, the activation of downstream DNMT3A caused by PPAR activation induced the methylated modification of inflammatory gene promoter sites, resulting in blocked binding of TFs to the promoters (see Figure 3). Therefore, PPAR activation is essential for the anti-inflammatory effect of galangin, while DNMT3A activation plays a supporting role. These findings could explain why GW9662 and DNMT3A reverse the protective effect of galangin to varying degrees.

As shown in Figure 3, there are at least two mechanisms involved in the anti-inflammatory effect caused by PPAR stimulation. Firstly, PPAR activation could directly transmit a transcription factor (TF) inhibitory signal, resulting in inhibition of TF synthesis for inflammatory genes. Secondly, the excited PPAR could further activate the nuclear methyltransferase (like DNMT3A), which promoted the methylation of CpG island at the promoter site of the inflammatory gene, thereby interfering the binding of TFs to the promoter sites. Under the abovementioned mechanisms, galangin eventually inhibited the synthesis of inflammatory mediators induced by LPS and alleviated the inflammatory damage.

## 5. Conclusions

This study is the first to prove that promoting methylation modification is part of the anti-inflammatory mechanism of galangin. Animal disease models further confirmed the effectiveness and safety of galangin in inhibiting inflammatory response and injury. However, the research results still have some limitations. First of all, regarding the anti-inflammatory mechanism related to methylation, DNMT3A, which widely exists in the biosphere, should regulate the expression of the CpG island gene in the intracellular promoter. After being activated by the PPAR agonist galangin, the mechanism of specific action on inflammatory target genes is still worth exploring. In addition, there is an urgent need to carry out clinical trials of galangin. It is hoped that the drug will help to overcome human inflammatory diseases as soon as possible.

## Figures and Tables

**Figure 1:** PPAR/DNMT3A pathway mediates the inhibition of inflammatory molecule synthesis by galangin in rat monocytes. (a) The WB assay results of PPAR and DNMT3A contents in BALF monocyte nuclei for various groups. (b, c) The relative levels of PPAR and DNMT3A expression, respectively. (d) The WB assay results of p65 and AP-1 levels in BALF monocyte nuclei. (e) The relative levels of p65 and AP-1 expression. In all the abovementioned analyses, *β*-actin is used as the internal control. (g, i) The blue parts present the CpG islands located in the promoter regions of rat IL-6 and TNF-a, respectively. There are binding sites for corresponding TFs within the aforementioned CpG islands, and the Chip-qPCR amplification regions are also located in these islands. (h) The Chip-qPCR results of phosphorylated p65 bound to the CpG island in the IL-6 promoter, where the relative density of bands in the upper gel electrophoresis map represents the semiquantitative PCR result. As is clear, the size of the amplification region at the IL-6 promoter site is 275 bp, and the reference sequence is the second intron region of IL-6, which has a size of 158 bp. Meanwhile, the bar graph describes the relative binding capacity of p65 that was analyzed by AlphaEase FC version 4. (j) The Chip-qPCR results shows AP-1 binding to the CpG island in the TNF-a promoter, where the amplification region has a size of 338 bp. The bar graph describes the relative binding capacity of AP-1, and the reference sequence is the same as that used in the IL-6 assay. ^*∗*^*P* < 0.05 versus Sham group; ^*∗∗*^*P* < 0.05 versus LPS group; ^#^*P* < 0.05 versus LPS + GAL group; ^##^*P* < 0.05 versus LPS + GAL and LPS + GAL + GW9662 groups.

**Figure 2:** Galangin attenuates LPS-induced lung injury, while GW9662 and DNMT3A interferences reverse this effect. (a, b) The concentrations of IL-6 and TNF-a in BALF for various groups, respectively. (c) Comparison of the dry/wet weight ratios of lung tissues among groups. (d) The HE staining observations of rat lung tissues for various treatment groups under a light microscope. (e) The time-varying Kaplan–Meier survival curves of SD rats in various groups. ^*∗*^*P* < 0.05 versus Sham group; ^*∗∗*^*P* < 0.05 versus LPS group; ^#^*P* < 0.05 versus LPS + GAL group; ^##^*P* < 0.05 versus LPS + GAL and LPS + GAL + GW9662 groups.

**Figure 3:** Molecular mechanisms of anti-inflammatory effect for PPAR agonist galangin.

**Table 1:** Sequences related to amplified IL-6 and TNF-a promoter regions (including TF binding sites) and the reference sequence.

	Position (distance from TSS)	Sequence information	PCR primer
IL-6 promotor	−632 ⟶ −358	aa**ggagacac**gagacgaag........	F:5′-aa**ggagacac**gagacgaag-3′
		p65	
		..............g**tattgtg**tacgttgctta	R:5′-attcgttgc**atgtgtatg**-3′
		p65	

TNF-a promotor	−656 ⟶ −319	aagcga**attctcag**acgcagcca........	F:5′-ctcc**attctcag**acgcagcca-3′
		AP-1	
		......**gtctaagt**ctcccgcctac	R:5′-catccgccctc**gtctaagt**-3′
		AP-1	

Reference sequence (IL-6 intron)	74 ⟶ 231	tccattcattctctttgctcctg...............	F:5′-tccattcattctctttgct-3′
		.............tctattcacagtggacacaatta	R:5′-ttcacagtggacacaatta-3′

*Note.* Bold parts indicate the TF binding sites.

## Data Availability

The data underlying the results presented in the study are included within the manuscript.

## References

[1] Habashi N. M., Camporota L., Gatto L. A., Nieman G. (1985). Functional pathophysiology of SARS-CoV-2-induced acute lung injury and clinical implications. *Journal of Applied Physiology*.

[2] Zhao F. C., Guo K. J., Li Z. R. (2013). Osteonecrosis of the femoral head in SARS patients: seven years later. *European Journal of Orthopaedic Surgery and Traumatology*.

[3] Sok S. P. M., Ori D., Wada A. (2021 Jun 18). 1’-Acetoxychavicol acetate inhibits NLRP3-dependent inflammasome activation via mitochondrial ROS suppression. *International Immunology*.

[4] Yi Y. S. (2018 Jul). Regulatory roles of flavonoids on inflammasome activation during inflammatory responses. *Molecular Nutrition & Food Research*.

[5] Xu L. J., Yu M. H., Huang C. Y. (2018). Isoprenylated flavonoids from Morus nigra and their PPAR*γ* agonistic activities. *Fitoterapia*.

[6] Jiang Z., Sang H., Fu X., Liang Y., Li L. (2015). Alpinetin enhances cholesterol efflux and inhibits lipid accumulation in oxidized low-density lipoprotein-loaded human macrophages. *Biotechnology and Applied Biochemistry*.

[7] He X., Wei Z., Wang J. (2016). Alpinetin attenuates inflammatory responses by suppressing TLR4 and NLRP3 signaling pathways in DSS-induced acute colitis. *Scientific Reports*.

[8] Han M., Gao H., Ju P. (2018). Hispidulin inhibits hepatocellular carcinoma growth and metastasis through AMPK and ERK signaling mediated activation of PPAR*γ*. *Biomedicine & Pharmacotherapy*.

[9] Hu K., Yang Y., Tu Q., Luo Y., Ma R. (2013). Alpinetin inhibits LPS-induced inflammatory mediator response by activating PPAR-*γ* in THP-1-derived macrophages. *European Journal of Pharmacology*.

[10] Ghizzoni M., Haisma H. J., Maarsingh H., Dekker F. J. (2011). Histone acetyltransferases are crucial regulators in NF-*κ*B mediated inflammation. *Drug Discovery Today*.

[11] Zhang Q., Zhao K., Shen Q. C. (2015). Tet2 is required to resolve inflammation by recruiting Hdac2 to specifically repress IL-6. *Nature*.

[12] Zampetaki A., Xiao Q., Zeng L., Hu Y., Xu Q. (2006). TLR4 expression in mouse embryonic stem cells and in stem cell-derived vascular cells is regulated by epigenetic modifications.TLR4 expression in mouse embryonic stem cells and in stem cell-derived vascular cells is regulated by epigenetic modifications.Biochem Biophys. *Biochemical and Biophysical Research Communications*.

[13] Wierda R. J., Rietveld I. M., van Eggermond M. C. (2015). Global histone H3 lysine 27 triple methylation levels are reduced in vessels with advanced atherosclerotic plaques. *Life Sciences*.

[14] Greißel A., Culmes M., Burgkart R. (2016). Histone acetylation and methylation significantly change with severity of atherosclerosis in human carotid plaques. *Cardiovascular Pathology*.

[15] Liang Y., Yang X. L., Ma L. N. (2013). Homocysteine-mediated cholesterol efflux via ABCA1 and ACAT1 DNA methylation in THP-1 monocyte-derived foam cells. *Acta Biochimica et Biophysica Sinica*.

[16] Bekkering S., Quintin J., Joosten L. A., van der Meer J. W., Netea M. G., Riksen N. P. (2014). Oxidized low-density lipoprotein induces long-term proinflammatory cytokine production and foam cell formation via epigenetic reprogramming of monocytes. *Arteriosclerosis, Thrombosis, and Vascular Biology*.

[17] Zhou C., Ye M., Ni S. (2018). DNA methylation biomarkers for head and neck squamous cell carcinoma. *Epigenetics*.

[18] Michailidi C., Theocharis S., Tsourouflis G. (2015). Expression and promoter methylation status of hMLH1, MGMT, APC, and CDH1 genes in patients with colon adenocarcinoma. *Experimental Biology and Medicine*.

[19] Sun P., Zhang S. J., Maksim S., Yao Y. F., Liu H. M., Du J. (2019). Epigenetic modification in macrophages: a promising target for tumor and inflammation-associated disease therapy. *Current Topics in Medicinal Chemistry*.

[20] Hu K., Liu L. J., Qian H. (2017). Alpinetin promotes the binding of PPAR and methyltransferase. *Xi Bao Yu Fen Zi Mian Yi Xue Za Zhi*.

[21] Tajima S., Suetake I., Takeshita K. (2016). Domain structure of the Dnmt1, Dnmt3a, and Dnmt3b DNA methyltransferases, 2016 [J]. *Advances in Experimental Medicine & Biology*.

[22] Seiler C. L., Fernandez J., Koerperich Z. (2018). Maintenance DNA methyltransferase activity in the presence of oxidized forms of 5-methylcytosine: structural Basis for TET-mediated DNA demethylation. *Biochemistry*.

[23] Hu K., Li Y., Liang M. (2019). Inhibitory effect of galangin on IL-6 expression by promoting cytosine methylation in CpG islands in the IL-6 promoter region. *Mol Genet Genomic Med*.

[24] Wan L. M., Meng D. M., Wang H. (2018). Preventive and therapeutic effects of thymol in a lipopolysaccharide-induced acute lung injury mice model. *Journal of Inflammation*.

[25] Bellani G., Laffey J. G., Pham T., Fan E, Brochard L, Esteban A (2016). Epidemiology, patterns of care, and mortality for patients with acute respiratory distress syndrome in intensive care units in 50 countries. *JAMA*.

